The article "Evaluation of Vertebral Function and Long-Term Quality of Life after Percutaneous Minimally Invasive Surgery in Patients with Thoracolumbar Spine Fractures" was retracted in 2023. Reasons: signs of a paper mill; suspected computer-generated content; unreliable results or conclusions; concerns about the data.

# Evaluation of Vertebral Function and Long-Term Quality of Life after Percutaneous Minimally Invasive Surgery in Patients with Thoracolumbar Spine Fractures

**DOI:** 10.1155/2022/2723542

**Published:** 2022-02-23

**Authors:** Bin Liu, QiaoHong Li, Hui Xie, XinPan Hu, XueKun Pan

**Affiliations:** Department of Emergency Trauma Surgery, First People's Hospital of Yunnan Province (the Affiliated Hospital of Kunming University of Science and Technology), Kunming, Yunnan 650032, China

## Abstract

**Objective:**

To investigate the changes in vertebral function after minimally invasive surgery in patients with thoracolumbar spinal fractures and investigate the impact of percutaneous minimally invasive surgery on patients' quality of life by following up the patients in the long term.

**Methods:**

A retrospective analysis was performed to select 80 patients with thoracolumbar spinal fractures treated in our hospital from April 2013 to October 2018, and the patients were divided into a study group and a control group according to the difference in their choice of procedure. The two groups were compared in terms of perioperative wound pain, serum creatine kinase (CK) activity, and C-reactive protein (CRP) levels, and the two groups were followed up for 2 years to compare the changes in anterior vertebral body height and Cobb's angle during the follow-up period and to compare the differences in quality of life between the two groups.

**Results:**

(1) The pain level of patients in the study group was significantly lower than that of the control group at the 1st and 3rd postoperative days (*p* < 0.05). (2) The CK activity and CPR level of patients in the study group were significantly lower than that of the control group at the 1st and 3rd postoperative days (*p* < 0.05). (3) Compared with the preoperative period, the height of the anterior border of the vertebral body and the Cobb's angle in both groups showed significant changes at 7 d, 6 months, one year, and two years after surgery (*p* < 0.05), suggesting that both procedures can significantly restore the height of the injured vertebra and improve the function of the vertebral body. (4) The somatic, physical, and psychological functions of patients in the study group were significantly greater than those in the control group at 6 months postoperatively (*p* > 0.05).

**Conclusion:**

Compared to traditional open surgery, minimally invasive percutaneous surgery for thoracolumbar fractures can significantly reduce perioperative pain and improve perioperative stress in patients, while achieving better surgical outcomes and a significantly improved quality of life in patients at long-term follow-up.

## 1. Introduction

The spine, also known as the spinal column, is a tissue made up of 26 vertebrae and one caudal vertebra, united by ligaments, joints, and intervertebral discs [1]. The spine supports the trunk, protects the internal organs, protects the spinal cord, and performs locomotion. The spine contains a top-down longitudinal spinal canal that contains the spinal cord [2]. In recent years, China's continual expansion of industrial construction and traffic vision has resulted in a considerable increase in the occurrence of various sorts of spine injuries. According to studies, the spine's stability is often compromised after thoracolumbar fractures, resulting in a high disability rate and a significant impact on patients' lives. As a result, aggressive surgical treatment is recommended to improve the stability of the fractured vertebrae and maximize the restoration of patients' ability to live [3, 4]. Traditional thoracolumbar fracture surgery is primarily performed through open surgery with the placement of pedicle screws, which has been shown to be highly invasive, with high bleeding and long postoperative hospital stays, and studies have also shown that patients frequently suffer from intractable low back pain or stiffness after surgery due to extensive stripping and stretching of muscles, fascia, and ligaments, which has a negative impact on their quality of life. [5, 6]. One of the most important research directions is the hunt for a less intrusive method. Mager was the first to use the percutaneous pedicle screw technique to treat spinal damage in 1982, paving the way for minimally invasive spine surgery. Long-term follow-up of percutaneous minimally invasive treatment of thoracolumbar spine fractures, on the other hand, has received little attention. In this study, we suggest setting up a control group to examine the feasibility of employing percutaneous minimally invasive surgery in thoracolumbar spine fractures in order to give a clinical reference for improving these patients' prognosis.

The article "Evaluation of Vertebral Function and Long-Term Quality of Life after Percutaneous Minimally Invasive Surgery in Patients with Thoracolumbar Spine Fractures" was retracted in 2023. Reasons: signs of a paper mill; suspected computer-generated content; unreliable results or conclusions; concerns about the data.

## 2. Materials and Methods

### 2.1. The General Materials

A retrospective analysis was performed on 80 patients with thoracolumbar spinal fractures who were treated in our institution between April 2013 and October 2018, and they were split into a study group and a control group based on the difference in surgery decision. Gender, age, weight, BMI, cause of injury, and fracture segment were included in the baseline clinical data and compared between the two groups; the results showed no statistically significant differences between the groups in terms of the above data (*p* > 0.05), implying that the two groups were comparable. See Table 1 for further information.

The following are the inclusion criteria: (1) patients who were diagnosed with thoracolumbar fractures by imaging and underwent internal fixation with pedicle screws; (2) age ≤ 55 years; and (3) the research process and method approved by the hospital's ethics committee and agreed to be performed.

The following are the exclusion criteria: (1) patients with comorbid psychiatric disorders; (2) those with ≥50% spinal canal occupancy and neurological impairment; (3) those with severe injury to the posterior longitudinal ligament complex; (4) those with intraoperative bone grafting or disc fusion; (5) those with comorbid systemic diseases or acute and chronic infections; (6) those with a history of previous thoracolumbar fractures or paravertebral drug treatment; (7) those with old fractures, osteoporotic fractures, or pathological fractures; (8) those who were lost during the study; (9) those who died during the study; and (10) those who had broken nails or rods during the study resulting in secondary surgery.

### 2.2. Intervention Methods

In preoperative preparation, patients in both groups underwent preoperative imaging as soon as possible to exclude contraindications to surgery and to arrange early surgery.

In the control group, the patient was placed in a prone position with the thorax and abdomen suspended. After general anaesthesia, a median longitudinal incision was made behind the spine with the diseased vertebral body as the centre, fully exposing the base of the transverse processes of one vertebral body above and below the diseased vertebral body and the upper and lower articular processes. The bone cone is turned into the arch at an angle of 12-15° to the sagittal plane (maximum depth of 4 cm), the hole is tapped, and the appropriate length of arch nail is inserted (the remaining 3 nails are placed in the same manner as above).

The patient in the research was treated in a prone hyperextended posture with the abdomen hanging in the air by percutaneous minimally invasive surgery. After fluoroscopy has determined that the puncture needle has not breached the medial cortex, a lateral fluoroscopic view is obtained, and the needle is determined to be parallel to the endplate once more, the puncture is performed to 0.5-1.0 cm anterior to the posterior edge of the vertebral body, the core is withdrawn and a guide wire is placed, the puncture needle is removed, and the canal and protective cannula are expanded in turn through the guide wire and the pedicle (the remaining three pedicle nails are placed in the same way). The remaining three pedicle screws are installed in the same manner. Finally, a rod device is placed and the incision is closed with sutures under fluoroscopy after repositioning to a satisfactory position.

The article "Evaluation of Vertebral Function and Long-Term Quality of Life after Percutaneous Minimally Invasive Surgery in Patients with Thoracolumbar Spine Fractures" was retracted in 2023. Reasons: signs of a paper mill; suspected computer-generated content; unreliable results or conclusions; concerns about the data.

### 2.3. Observation Indicators and Assessment Criteria

#### 2.3.1. Perioperative Pain Level

A visual analogue scale (VAS) [7] was used to assess the pain level of the two groups of patients before surgery, at the first postoperative day, at the third postoperative day, and at the fifth postoperative day and to compare the differences between the groups.

#### 2.3.2. Perioperative Serum Creatine Kinase Activity and C-Reactive Protein Level

Fasting elbow venous blood samples were collected from patients in both groups before surgery, on the 1st day postoperatively and on the 3rd day postoperatively, respectively, and the serum was retained after centrifugation, and the levels of CK and CRP were measured by enzyme-linked immunosorbent assay (ELISA) and chemical immunoassay, and the differences between the groups were compared.

#### 2.3.3. Follow-Up of Anterior Vertebral Body Margin Height and Cobb's Angle in Both Groups

Patients in both groups were followed up for a period of 2 years, and the anterior vertebral body height and Cobb's angle were recorded before, 7 d after, 6 months after, 1 year after, and 2 years after surgery. The height of the anterior vertebral body = (actual height of the anterior border of the injured vertebra/reference height of the anterior border of the injured vertebra) × 100% [8]. Cobb's angle was measured as follows: the vertical lines of the superior vertebral body and the inferior vertebral body of the injured vertebra were made on the lateral radiographs, and the angle between the two vertical lines was Cobb's angle [9].

#### 2.3.4. Quality of Life at Follow-Up

The SF-36 was used to assess the quality of life of both groups at 6 months after surgery. The SF-36 can be divided into three main dimensions: physical function, physiological function, and psychological function, with higher scores in each dimension representing better quality of life.

### 2.4. Statistical Methods

The data were entered into Excel 2019, and SPSS 22.0 statistical software was selected for statistical analysis of the collected data. Count data were expressed using *n* (%), a chi-square test was selected for comparison of differences between groups, mean ± standard deviation was selected for measurement data, an independent sample *t*-test was selected for comparison of differences between groups, and a paired sample *t*-test was selected for comparison of before and after continuous variables. *p* < 0.05 was taken as the difference was statistically significant [10].

## 3. Results

### 3.1. Comparison of Wound Pain in the Two Groups

The comparison showed that the difference in pain level between the two groups was not statistically significant before surgery (*p* > 0.05), and the pain level of the patients in the study group was significantly lower than that of the control group at the 1st and 3rd postoperative days (*p* < 0.05). See Table 2 and Figure 1.

The article "Evaluation of Vertebral Function and Long-Term Quality of Life after Percutaneous Minimally Invasive Surgery in Patients with Thoracolumbar Spine Fractures" was retracted in 2023. Reasons: signs of a paper mill; suspected computer-generated content; unreliable results or conclusions; concerns about the data.

### 3.2. Comparison of Serum Creatine Kinase Activity and C-Reactive Protein Levels between the Two Groups of Patients

Serum CK activity and CRP levels were measured in the blood samples collected from the two groups before surgery, at the first day and the third day after surgery, respectively (control group (*p* < 0.05)). See Table 3 and Figure 2.

### 3.3. Analysis of Changes in Anterior Vertebral Body Height and Cobb's Angle in the Two Groups

The anterior margin height and Cobb's angle of the vertebral body in both groups were measured before surgery, 7 days after surgery, 6 months after surgery, 1 year after surgery, and 2 years after surgery, and imaging examinations were performed before surgery, 7 days after surgery, 6 months after surgery, 1 year after surgery, and 2 years after surgery. There was no statistically significant difference between the two groups (*p* > 0.05). According to the results, both procedures successfully restored the height and function of the afflicted spine.

At the postoperative observation time point, there was no statistically significant difference between the groups in terms of anterior vertebral height and Cobb's angle (*p* > 0.05).  Figure 3 shows the situation.

### 3.4. Comparison of Postoperative Quality of Life between the Two Groups

At 6 months postoperatively, the SF-36 scale was used to measure the quality of life of the two groups of patients, and the differences between the groups were compared in terms of the scale's scores on each dimension.  Figure 4 shows the situation.

## 4. Discussion

Thoracolumbar spine fractures (T11-L2) are those that occur in the thoracic 11-lumbar 2 (T11-L2) stage of the spine [11]. As incidents such as traffic accidents and industrial injuries continue to rise in China, the frequency of spinal fractures in the thoracolumbar area has also increased significantly [12]. Compression of the spinal cord can easily injure the cauda equina, resulting in sensory impairment in moderate instances or paralysis and loss of movement in severe cases, lowering the patient's quality of life [13]. Early surgical treatment is an important means of relieving spinal cord compression and reducing neurological impairment. Decompression by incision and fixation of the vertebrae can minimise spinal cord compression and improve the patient's mobility [14].

The typical thoracolumbar fracture method is primarily open surgery, which is becoming less popular because of the evident trauma and the patient's extended postoperative recovery period. Percutaneous lumbar pedicle screw fixation under X-ray guidance was first described by Mathews et al. in 1995, pioneering the method of percutaneous pedicle screw fixation [15]. Percutaneous pedicle screw treatment has been found to have a good stabilizing effect in patients, correcting vertebral instability owing to fracture and enhancing vertebral function [16].

The article "Evaluation of Vertebral Function and Long-Term Quality of Life after Percutaneous Minimally Invasive Surgery in Patients with Thoracolumbar Spine Fractures" was retracted in 2023. Reasons: signs of a paper mill; suspected computer-generated content; unreliable results or conclusions; concerns about the data.

In this study, a controlled group was set up to investigate how percutaneous minimally invasive intraspinal nailing of patients with thoracolumbar fractures could significantly improve perioperative pain and stress compared to traditional open surgery. It has been pointed out that surgery is a special form of trauma to the body, causing local tissue damage and organ dysfunction, and it has been a research direction for surgeons to minimise the perioperative stress response of patients [17]. In this paper, serum CK and CRP levels were significantly lower in the study group than in the control group from the first to the third postoperative day, which indicates that the postoperative stress response was more moderate in the study group than in the control group, suggesting that the patients in the study group were less traumatized, and analyzing this is also an important reason for the lower VAS scores in the study group during the perioperative period.

After a long period of time, the differences in anterior vertebral margin height and Cobb's angle between the two groups were not statistically significant, but there were significant differences in anterior vertebral margin height and Cobb's angle between the two groups at intra- and postoperative comparison, indicating that both techniques were effective in alleviating the fracture symptoms in the patients. When 100 patients with thoracolumbar fractures were observed in a clinical setting, it was shown that patients who had minimally invasive surgery had greater vertebral function at 2 years of follow-up compared to those who underwent open surgery [18, 19]. In the long run, this might have an effect on the function of the vertebral body. Percutaneous minimally invasive surgery has several advantages over traditional open surgery, according to the findings of this study: the needle-guiding technique increases the accuracy of spiral nail placement, less muscle stripping during surgery, less trauma to the patient, and better postoperative repositioning with less time in bed, all of which serve as practical references for the application of this procedure in clinical practice. In conclusion, compared to traditional open surgery, percutaneous minimally invasive surgery in patients with thoracolumbar fractures can significantly alleviate perioperative pain symptoms and improve their perioperative stress status, while at long-term follow-up patients can achieve better surgical results and a significantly improved quality of life.

The article "Evaluation of Vertebral Function and Long-Term Quality of Life after Percutaneous Minimally Invasive Surgery in Patients with Thoracolumbar Spine Fractures" was retracted in 2023. Reasons: signs of a paper mill; suspected computer-generated content; unreliable results or conclusions; concerns about the data.

## Figures and Tables

**Figure 1:** shows a comparison of the two groups' wound pain levels. Before surgery, there was no statistically significant difference in pain levels between the two groups (*p* > 0.05), but pain levels in the study group were significantly lower than those in the control group on the 1st and 3rd postoperative days (*p* = 0.05), and the difference in pain levels between the two groups on the 5th postoperative day was not statistically significant (*p* = 0.05). # represents the difference between groups of the same index which was not statistically significant. # represents a statistically significant difference between groups comparing the same index.

**Figure 2:** Comparison of serum creatine kinase activity and C-reactive protein levels in the two groups. The differences in serum CK activity and CRP levels between the two groups before surgery were not statistically significant (*p* > 0.05), while the CK activity and CPR levels of patients in the study group were significantly lower than those of the control group at postoperative day 1 and postoperative day 3 (*p* < 0.05). # represents a statistically significant difference between groups for the same index.

**Figure 3:** Analysis of changes in anterior vertebral body margin height and Cobb's angle in the two groups. The differences in anterior vertebral body margin height and Cobb's angle between the two groups of patients at the preoperative and postoperative observation points were not statistically significant (*p* > 0.05). At 7 days postoperatively, 6 months postoperatively, 1 year postoperatively, and 2 years postoperatively, there were significant changes in the anterior vertebral body margin height and Cobb's angle in both groups compared to the preoperative period (*p* < 0.05).

**Figure 4:** Comparison of postoperative quality of life between the two groups of patients. The physical, physiological, and psychological functions of the patients in the study group were significantly greater than those in the control group, and the difference between the groups was statistically significant (*p* < 0.05). ^#^The difference between groups was statistically significant.

**Table 1:** Comparison of general clinical indicators between the two groups ($\bar{x}\pm s$)/[*n*(%)].

General clinical information		Research group (*n* = 40)	Control group (*n* = 40)	*t*/*X*^2^	*p*
Gender	Male	25	26	0.005	0.945
	Female	15	14		
Average age (years)		41.11 ± 3.28	41.21 ± 3.34	0.106	0.781
Average weight (kg)		65.18 ± 3.91	65.31 ± 3.77	0.119	0.780
Average BMI (kg/m^2^)		20.19 ± 2.19	19.98 ± 2.28	0.331	0.724
Cause of injury	Traffic accidents	15	14	0.889	0.231
	Falling injuries	14	13		
	Heavy object injuries	7	10		
	Injuries from falls	4	3		
Fractured segments	T11	8	7	0.891	0.221
	T12	9	8		
	L1	7	10		
	L2	10	10		
	L3	6	5		

The article "Evaluation of Vertebral Function and Long-Term Quality of Life after Percutaneous Minimally Invasive Surgery in Patients with Thoracolumbar Spine Fractures" was retracted in 2023. Reasons: signs of a paper mill; suspected computer-generated content; unreliable results or conclusions; concerns about the data.

**Table 2:** Comparison of perioperative pain levels between the two groups ($\bar{x}\pm s$).

Group	Number of examples	Preoperative	1st postoperative	3rd postoperative	5th postoperative
Research groups	40	6.44 ± 1.29	3.28 ± 0.87^#^	1.29 ± 0.21^#^	0.34 ± 0.09^#^
Control group	40	6.51 ± 1.19	4.38 ± 0.97^#^	2.21 ± 0.45^#^	0.35 ± 0.10^#^
*t*	—	0.252	5.339	11.717	0.47
*p*	—	0.802	<0.001	<0.001	0.64

Compared to preoperative, ^#^*p* < 0.05.

**Table 3:** Comparison of serum CK activity and CRP levels between the two groups ($\bar{x}\pm s$).

Group	Number of examples	CK (IU/L)			CRP (mg/L)		
		Preoperative	1st postoperative	3rd postoperative	Preoperative	1st postoperative	3rd postoperative
Research group	40	95.58 ± 10.22	200.12 ± 23.39^#^	140.39 ± 20.11^#^	2.39 ± 0.98	10.28 ± 1.98^#^	9.21 ± 1.22^#^
Control group	40	96.29 ± 9.89	340.11 ± 20.39^#^	180.29 ± 19.89^#^	2.41 ± 0.78	13.29 ± 2.01^#^	10.58 ± 1.01^#^
*t*	—	0.316	28.533	8.922	0.101	6.747	5.471
*p*	—	0.753	<0.001	<0.001	0.92	<0.001	<0.001

Compared to preoperative, ^#^*p* < 0.05.

## Data Availability

The data used to support the findings of this study are included within the article.
